The article "2-Day versus C-reactive protein guided antibiotherapy with levofloxacin in acute COPD exacerbation: A randomized controlled trial" was retracted in 2024. Reasons: duplicate publication; lack of ethics approval or compliance; concerns about the data; concerns about the results or conclusions.

# 2-Day versus C-reactive protein guided antibiotherapy with levofloxacin in acute COPD exacerbation: A randomized controlled trial

**DOI:** 10.1371/journal.pone.0251716

**Published:** 2021-05-20

**Authors:** Msolli Mohamed Amine, Messous Selma, Sekma Adel, Bel haj ali Khaoula, Khalil Mohamed Hassene, Trabelsi Imen, Abdelghani Ahmed, Ben Brahim Nadia, Ben Dhaya Yosra, Razgallah Rabie, Grissa Mohamed Habib, Beltaief Kaouthar, Methamem Mehdi, Belguith Asma, Bouida Wahid, Boukef Riadh, Boubaker Hamdi, Nouira Semir, on behalf of the GREAT Network

**Affiliations:** 1 Emergency Department, Fattouma Bourguiba University Hospital, Monastir, Tunisia; 2 Research Laboratory LR12SP18, Monastir University, Monastir, Tunisia; 3 Pneumology Department, Farhat Hached University Hospital, Sousse, Tunisia; 4 Medis Laboratories, Tunis, Tunisia; 5 DACIMA Consulting, Tunis, Tunisia; 6 Emergency Department, Farhat Hached University Hospital, Sousse, Tunisia; 7 Department of Preventive Medicine, Fattouma Bourguiba University Hospital, Monastir, Tunisia; 8 Emergency Department, Sahloul University Hospital, Sousse, Tunisia; Prince Sattam Bin Abdulaziz University, College of Applied Medical Sciences, SAUDI ARABIA

## Abstract

**Introduction:**

Duration of antibiotic treatment in acute exacerbation of COPD (AECOPD) is most commonly based on expert opinion. Biomarker guided strategy is increasingly recommended to limit unnecessary antibiotic use. We performed a randomized controlled study to evaluate the efficacy of 2-day versus C-reactive protein (CRP)-guided treatment with levofloxacin in patients with AECOPD.

**Methods:**

Patients with AECOPD were randomized to receive oral levofloxacin daily for 7 days unless the serum CRP level decreased by at least 50% from the baseline value or levofloxacin for two days; thereafter, oral placebo tablet was prescribed according to the CRP. The primary outcome measure was cure rate, and secondary outcome included need for additional antibiotics, intensive care unit (ICU) admission, exacerbation rates and exacerbation free interval (EFI) within one-year follow-up.

**Results:**

In intention to treat (ITT) analysis, cure rate was 76.1% (n = 118) and 79.3% (n = 123) respectively in 2-day and CRP-guided groups. In per protocol (PP) analysis, cure rate was 73% (n = 92) and 70.4% (n = 88) respectively in 2-day and CRP-guided groups. The difference between the two groups was not significant. The need for additional antibiotics and ICU admission rates were not significantly different between the two groups. One-year exacerbation rate was 27% (n = 42) in 2-day group versus 30.3% (n = 47) in CRP-guided group (p = 0.53); the EFI was 125 days (interquartile range, 100–151) versus 100 days (interquartile range, 78–123) in 2-day and CRP-guided groups respectively (p = 0.45). No difference in adverse effects was detected.

The article "2-Day versus C-reactive protein guided antibiotherapy with levofloxacin in acute COPD exacerbation: A randomized controlled trial" was retracted in 2024. Reasons: duplicate publication; lack of ethics approval or compliance; concerns about the data; concerns about the results or conclusions.

**Conclusion:**

Levofloxacin once daily for 2 days had similar efficacy compared to CRP-guided in AECOPD. This short course treatment decreased antibiotic consumption which would improve patient compliance and reduce adverse effects.

## Introduction

Chronic obstructive pulmonary disease (COPD) is a common disease worldwide and a leading cause of death and disability globally [1–3]. Given that bacteria are implicated in a substantial proportion of acute exacerbation of COPD (AECOPD), antibiotics are frequently used. However, this current practice may lead to antibiotic overuse further increasing drug resistance and side effects [4–10]. Implementing specific rules that reduce unnecessary antibiotherapy prescription and duration is highly beneficial [11,12]. Available studies showed that antibiotic treatment could be shortened and this could be achieved with or without the aid of biomarkers. Guidelines stated that antibiotic treatment should be maintained at an average of 7 to 10 days while some studies showed the non-clinical inferiority of courses as short as 3 days in many specific diseases like respiratory infections and AECOPD [13–15]. C-reactive protein (CRP) is an acute phase protein that rises rapidly in infections and is considered a useful biomarker to guide antibiotherapy in AECOPD [16–18]; however, there was no trials comparing clinical effectiveness and cost-effectiveness of CRP-guided strategy and a fixed short course of antibiotic in AECOPD patients. Hence, we conducted this study to compare the efficacy of a 2-day course of levofloxacin with CRP-guided antibiotic prescription in AECOPD.

## Materials and methods

### Study design

We conducted a prospective, randomized, double-blinded controlled study from May 2017 to January 2019 including patients with AECOPD admitted to the emergency department (ED). Fattouma Bourguiba university hospital ethic committee, Sahloul university hospital ethic committee and Farhat Hached university hospital ethic committee approved the study before implementation, and all included patients provided written informed consent. Also, the study protocol was prepared in accordance with the revised Helsinki Declaration for Biomedical Research Involving Human Subjects and Guidelines for Good Clinical Practice and was registered at www.clinicaltrials.gov: **NCT02067780.**

### Settings and participants

This study included adult patients admitted to three EDs (Fattouma Bourguiba University Hospital Monastir, Sahloul University Hospital Sousse, and Farhat Hached University Hospital Sousse). Patients were eligible for inclusion in the cohort if they were 45 years or older and had a clinical diagnosis of COPD defined according to the Global Initiative of Chronic Obstructive Lung Disease (GOLD). AECOPD was defined as a change in patients’ baseline dyspnea, cough, or sputum beyond day-to-day variability, sufficient to warrant a change in management other than optimization of bronchodilator therapy. Patients were excluded if they presented with one of the following conditions: clinical evidence of hemodynamic compromise with the need for vasoactive drugs, immediate need for mechanical ventilation, Glasgow coma scale <12, pneumonia, previous adverse reactions to the study drug, antibiotic treatment in the previous days, pregnancy or lactation, severe renal (creatinine clearance 40 mL/min) or hepatic impairment, or lung disease other than COPD that could affect the clinical evaluation of the treatments. Patients with active alcohol or drug abuse were also excluded.

The article "2-Day versus C-reactive protein guided antibiotherapy with levofloxacin in acute COPD exacerbation: A randomized controlled trial" was retracted in 2024. Reasons: duplicate publication; lack of ethics approval or compliance; concerns about the data; concerns about the results or conclusions.

### Randomization and intervention

For all included patients, demographic, clinical, and biological data were collected at baseline. These included the patients’ comorbidities, number of exacerbations in the past year, physical examination findings, blood gas analysis, and standard laboratory test results. Expectorated sputum samples were collected for pathogen culture, and all data were recorded in standardized electronic case report forms. Noninvasive ventilation (NIV) was performed for patients with an arterial carbon dioxide partial pressure >45 mmHg and pH <7.35, using supplemental oxygen to obtain a pulse oxygen saturation >90%. Patients were randomly assigned (1:1) to one of two treatment arms: (1) the intervention (CRP-guided) group: 500 mg (one tablet) of oral levofloxacin daily for 7 days unless the serum CRP level decreased by at least 50% from the baseline value. The serum CRP levels were measured at the ED admission on days 2, 4, and 6, and made available to the attending physicians. (2) The standard care (control) group: 500 mg of levofloxacin daily for the first two days; thereafter, the oral placebo tablet was prescribed according to the CRP values as in the CRP-guided group to maintain the blindness of the study. The randomization sequence was generated using a sealed envelope sequence generator stratified according to the investigator site. Online inclusion of patients according to the concealed sequence was performed with an independent, centralized web-based system (DACIMA Tunisia; https://www.dacimasoftware.com). Additionally, to ensure blinding, active drugs, as well as the placebo tablets, were encapsulated for identical appearance and placed in sealed envelopes. All patients who received at least one dose of the study medication comprised the intent-to-treat (ITT) population and were treated in the ED during the first 48 hours (h). Also, all patients received intravenous methylprednisolone (0.3 mg/kg every 6h), nebulized bronchodilator, and fluid therapy, while other medications were prescribed at the attending physician’s discretion. After 48-h ED stay, patients were discharged if their condition improved; otherwise, they were hospitalized in the ward or ICU if they required intubation or needed NIV. All the patients were monitored over seven days, adverse effects including photosensitivity, nausea, diarrhea, headache, tendinitis, tendon rupture, hyper-hypoglycemia, seizures, prolonged QT interval, and peripheral neuropathy, were reported and rated by the investigator as possibly, probably, or related to the study treatment. Long-term follow-up was made by phone contact on the 15th day of every month for 12 months after the study treatment. If the patient was not reachable, the next of kin and/or the patient’s general practitioner were contacted. Physicians who collected outcome data were not aware of the treatment allocation. The vital status, time to next acute exacerbation, and exacerbation-free interval (EFI) were recorded with each phone communication.

The article "2-Day versus C-reactive protein guided antibiotherapy with levofloxacin in acute COPD exacerbation: A randomized controlled trial" was retracted in 2024. Reasons: duplicate publication; lack of ethics approval or compliance; concerns about the data; concerns about the results or conclusions.

### Outcome analysis

Outcome analysis were performed on the intent-to-treat and per-protocol (PP) populations. Clinical cure rate was considered as the primary outcome. It was defined as resolution of acute signs and symptoms of AECOPD to baseline level (non-exacerbated state), together with resolution of fever if present at inclusion study entry and no reason for treatment failure. Secondary outcome included EFI, ICU admission rate, and need for additional antibiotics. The decision to initiate new antibiotics was left to the discretion of the treating physician. One-year exacerbation and death rates were considered as secondary outcome. The antibiotic sparing effect was also assessed; it was defined as the duration of levofloxacin treatment possibly saved with 2-day regimen compared to CRP-guided strategy.

#### Statistical analysis

The primary objective was to demonstrate that levofloxacin treatment for 2 days was non-inferior to CRP-guided treatment. Analysis at follow-up for the primary outcome was based on the ITT population and per-protocol (PP) population. Data from previous studies, used to estimate the frequency of the primary outcome of the present study, suggested that exacerbations within 1 year occurred in approximately 50% of the patients. To define the non-inferiority of the 2-day course compared to the CRP-guided treatment, we selected a 15% difference in the percentage of cure rate as a clinically tolerable upper limit. We hypothesized that cure rates for the two treatment plans would be equal (at 80%) and considered a difference of ≤15% to be irrelevant. Then, setting β = 0.20 and α = 0.05 (one-tail), the estimated sample size was 140 patients per arm. Taking into account an estimated 10% drop-out rate of patients at 6-month follow-up, we increased the sample size to 155 patients per arm. Qualitative data were described with frequencies and percentages; quantitative data were described with the mean ± standard error or with the median, interquartile interval, and range. Baseline characteristics of the patients were compared with the unpaired t-test or the Wilcoxon rank sum test for continuous variables, depending on their distributions. Percentage differences were compared using the Fisher’s exact test (or χ2 test, when appropriate). In case of skewed distributions, continuous variables were logarithmically transformed for further analysis. Comparisons of the incidence rates of AEs between the two study groups were performed descriptively. No interim analysis was planned or performed for this study. All statistical tests were two-sided and performed at a 0.05 significance level using the SPSS software, version 20.0.

The article "2-Day versus C-reactive protein guided antibiotherapy with levofloxacin in acute COPD exacerbation: A randomized controlled trial" was retracted in 2024. Reasons: duplicate publication; lack of ethics approval or compliance; concerns about the data; concerns about the results or conclusions.

## Results

A total of 500 patients were screened, and 310 patients were randomized (ITT population) to receive a 2-day course of levofloxacin (n = 155), or CRP-guided protocol (n = 155). The PP population comprised 251 patients at the end of follow-up with 126 and 125 patients, respectively, for the 2-day and CRP-guided groups (Fig 1). Main reason for withdrawing patients from the ITT analysis was incomplete (end-of therapy) evaluation (29 patients in 2-day group and 30 patients in CRP-guided group). A description of the baseline characteristics of the patients is given in Table 1. The two treatment groups had similar baseline demographics and clinical findings (Table 1), as well as similar severity criteria of the episode as assessed by the number of exacerbations during the previous year and according to the Anthonisen classification. The median duration of treatment in the CRP-guided group was 3.6 days (interquartile intervals: 3.0–3.9). The two treatment groups were similar in the number of pathogens isolated at pre-therapy (52 versus 47, respectively, in the 2-day and CRP-guided groups). Haemophilus influenzae and chlamydophila pneumoniae which were isolated respectively from 18 and 15 patients, were the most common pathogens found (Table 2). CRP decreased significantly in the two groups over time compared to baseline values; this decrease was comparable between groups (Fig 2).

The article "2-Day versus C-reactive protein guided antibiotherapy with levofloxacin in acute COPD exacerbation: A randomized controlled trial" was retracted in 2024. Reasons: duplicate publication; lack of ethics approval or compliance; concerns about the data; concerns about the results or conclusions.

**Fig 1:** Flow chart.

**Fig 2:** C-reactive protein values at baseline and day 2, 4 and 6. CRP: C-reactive protein.

**Table 1:** Patients’ demographic and clinical characteristics at admission*.

	2-day group n = 155	CRP-guided group n = 155	p-value
Age years, mean (SD)	68.5±10.1	66.7±10.5	0.12
Sex ratio M/F	131/21	135/20	0.81
Smoking (pack-years), mean (SD)	53.4±13.2	67.2±15.6	0.15
Peak Expiratory Flow (L/min), mean (SD)	62.6±15.9	64.4±18.6	0.12
Body mass index (kg.m^2^), mean (SD)	26.8±7.5	26.4±4.5	0.62
Exacerbations within the past year, mean (SD)	2.1±1.8	2.4±1.9	0.11
**Past medical history n (%)**			
Hypertension	45(29)	48(30.9)	0.76
Heart failure	8(5.16)	1(0.64)	0.01
Diabetes	21(13.5)	27(17.4)	0.39
**Anthonisen classification n (%)**			
Type 1	34(21.9)	40(25.8)	0.42
Type 2	121(78.1)	115(74.2)	
**Blood pressure**			
Systolic mmHg, mean (SD)	138.2±29.1	136.2 ±25.2	0.54
Diastolic mmHg, mean (SD)	76.7±24.4	71.1±21.3	0.03
**Temperature (°C), mean (SD)**	37.1±0.8	37.0±0.5	0.47
**Pulse rate (b/min), mean (SD)**	105.3±23.1	106.7± 25.7	0.64
**Respiratory rate (c/min), mean (SD)**	26.4±5.4	26.3±8.6	0.9
**Blood gas**			
pH, median (IQR)	7.33(7.31–7.36)	7.32(7.30–7.36)	0.11
PaCO_2_ (mmHg), median (IQR)	41.9(39.9–45.5)	44.1(40.9–47.3)	0.5
**White blood cells (x 10**^**3**^**/mm**^**3**^**)**	13.35±11.12	12.83±4.97	0.61
**C-reactive protein (mg/L), median (IQR)**	60.61(45.12–76.11)	51.88(40–63.77)	0.37
**Median duration of therapy, median (IQR)**	2	3.6 (3–3.9)	0.19

* Intention-to-treat population.

Abbreviations: M/F: Male/female; IQR: Interquartile range.

**Table 2:** Bacteriologic results.

	2-day group	CRP-guided group
*Branhamella catarrhalis*	5	4
*Escherichia coli*	1	3
*Haemophilus influenzae*	10	8
*Haemophilus parainfluenzae*	1	4
*Klebsiella pneumoniae*	3	0
*Proteus mirabilis*	1	0
*Pseudomonas aeruginosa*	7	4
*Branhamella catarhalis*	6	4
*Providencia*	0	1
*Acinetobacter spp*	1	2
*Mycoplasma pneumoniae*	1	3
*Acinetobacter baumanni*	4	1
*Chlamydophila pneumoniae*	8	7
*Coxiella burnetii*	4	6
Total	52	47

Clinical outcomes for the ITT and PP populations showed that a 2-day regimen of levofloxacin was non-inferior to a CRP-guided strategy (Table 3). In ITT population, cure rate was similar in the 2 groups [76.1% and 79.3% in the 2-day group and CRP-guided group respectively; HR 1.46; 95% CI, 0.83 to 2.59; p = 0.49]. In PP population, cure rate was 73% and 70.4% in the 2-day group and 7-day group respectively (HR 1.00; 95% CI, 0.66 to 1.50; p = 0.65).

**Table 3:** Patients’ outcome.

	2-day group n = 155	CRP-guided group n = 155	P value	HR (95% CI)
**Primary Outcome**				
Cure rate, n (%)				
ITT	118(76.1)	123(79.3)	0.49	1.46(0.83–2.59)
PP	92(73.0)	88(70.4)	0.65	1.00(0.66–1.50)
**Secondary outcomes**				
Need for Additional Antibiotic Therapy, n (%)				
ITT	18 (11.6)	14(9)	0.45	1.04(0.54–2.00)
PP	12(9.5)	10(8)	0.67	1.42(0.74–2.72)
ICU Admissions, n (%)				
ITT	10(6.4)	11(7)	0.82	0.79(0.35–1.77)
PP	6(4.7)	8(6.4)	0.57	1.10(0.49–2.45)
Exacerbation free interval days, median (IQR)				
ITT	125(100–151)	100(78–123)	0.45	1.001(0.99–1.004)
PP	125(100–151)	99(76–121)	0.42	1.001(0.99–1.004)
One-year mortality, n (%)				
ITT	12(7.7)	7(4.5)	0..23	3.15(1.82–5.45)
PP	12(9.5)	7(5.6)	0.24	3.15(1.82–5.45)
One-year exacerbation rate, n (%)				
ITT	42(27)	47(30.3)	0.53	49.45(15.67–156.54)
PP	42(33.3)	47(37.6)	0.48	49.45(15.67–156.54)

Abbreviations: ITT intention-to-treat population; PP per-protocol population (2-day group n = 126; CRP- guided group n = 125); ICU intensive care unit.

The article "2-Day versus C-reactive protein guided antibiotherapy with levofloxacin in acute COPD exacerbation: A randomized controlled trial" was retracted in 2024. Reasons: duplicate publication; lack of ethics approval or compliance; concerns about the data; concerns about the results or conclusions.

### Secondary outcome

Data regarding secondary outcome in ITT population are shown in Table 3. Rate of additional antibiotic prescriptions was similar in the two groups [11.6% and 9% in the 2-day group and CRP-guided group respectively; (p = 0.45)]. ICU admission rate was 6.4% in the 2-day group and 7% in the CRP-guided group (p = 0.82). One-year exacerbation rate was not significantly different between the 2 groups (27% versus 30.3% in the 2-day group and CRP-guided group respectively; (p = 0.53). EFI was similar in the two treatment groups [125 days (interquartile range 100–151) versus 100 days (interquartile range 79–123) in the 2-day and CRP-guided groups respectively; p = 0.45]. The net antibiotic sparing effect with the 2 days levofloxacin fixed dose ranged from 1 to 2 days (median = 1.6 days).

### Safety

AEs were reported in one patient in the 2-day group. The incidence of AEs was very low in this study, with only one patient in the 2-day group; however, this was mild and did not require discontinuation of the treatment study.

## Discussion

Our results showed that in patients admitted with AECOPD, a 2-day course of levofloxacin was not clinically inferior to CRP-guided treatment in terms of cure rate, need for additional antibiotics, ICU admission, exacerbation free interval, and one-year exacerbation rate.

Inappropriate antibiotic use is frequent and represents the main risk factor for bacterial resistance. In this regard, reducing unnecessary prescription of antibacterial agents play a crucial role to maintain antibiotic effectiveness. Shortening antibiotic therapy duration could be one method to limit this increasing challenge, provided the clinical efficacy is not impaired. Previous studies have been performed to evaluate this possibility in AECOPD [19]. Stolbrink et al. conducted a meta-analysis, including 10 randomized controlled trials in which short and standard courses of antibiotics belonging to the same classes were compared [20]. Three of the studies involving fluoroquinolones were in favor of short-course treatment. Overall, the typical administration periods range from 5 to 14 days, but the evidence regarding the ideal index duration for antibiotics is limited. Several well-designed trials found that biomarker-based guidance in the treatment of AECOPD reduced the use of antibiotics with no apparent harm to patients [12]. Increasing data support the use of CRP and procalcitonin (PCT) treatment algorithms as an evidence-based approach to more individualized and judicious use of antibiotics in AECOPD [16,21]. One study has demonstrated that AECOPD patients admitted to the hospital with CRP ≥50 mg/L possibly benefitted more from antibiotics than patients with low CRP values [22]. Similar results were found in another study using a cutoff point of 40 mg/L [23]. In a recent multicenter, open-label, randomized, controlled trial conducted in the UK and Wales, Butler et al. showed that for patients with CRP <20 mg/L, antibiotics were unlikely to be beneficial and, in contrast, for those with a CRP >40 mg/L, antibiotics were likely to be beneficial [17]. Interestingly, almost all of our patients had a CRP level >40 mg/L and using CRP-guided strategy was associated with a reduction of antibiotic therapy duration to 3.6 days compared to the 7 to 10 day-regimen currently recommended. However, this duration is still higher than 2-day course which is found to be as effective. This means that CRP-guided strategy is useful to reduce antibiotic prescription but not sufficiently sensitive to titrate treatment duration. We estimate that 2 days could be the lowest effective antibiotic course in AECOPD and could be recommended to decrease the emergence of antimicrobial resistance and minimize costs. The effectiveness of such a short course of antibiotics means that the early infection period is the most sensitive to antibiotic effects, allowing a maximum decrease in the bacterial growth and for the immune system to gain time to acquire an enhanced ability to fight the microorganism [24]. Our findings also suggest that sterility of the infection site is not necessary for clinical healing and that the dogma that stopping antibiotic treatment early encourages resistance to antibiotics is not evidence-based [25]. Bacterial resistance due to post-antibiotic effect (PAE) is another potential factor that sustains the effectiveness of short antibiotic courses [26]. It refers to the suppression of bacterial growth, which persists after brief exposure of organisms to antimicrobials. Similar to aminoglycosides, fluoroquinolones have concentration-dependent bactericidal activity and prolonged PAE [27]. However, the exact duration of the PAE, which is also species-dependent, is unknown.

The article "2-Day versus C-reactive protein guided antibiotherapy with levofloxacin in acute COPD exacerbation: A randomized controlled trial" was retracted in 2024. Reasons: duplicate publication; lack of ethics approval or compliance; concerns about the data; concerns about the results or conclusions.

The main strength of our study is that it was double-blinded, which is not common in trials using a biomarker algorithm. Hospital staff and investigators were blinded to the randomization results, allowing for a low risk of performance bias. Also, this was a multicentric study, conducted over three years and covering all the four seasons, with minimal loss to follow up.

Our findings must be interpreted in the context of several potential limitations. First, since we only used levofloxacin in this study, it is uncertain if similar results would be obtained in response to other antibiotics. Therefore, extrapolating our results to other antibiotic classes is presumptive. Furthermore, patients with hemodynamic or respiratory instability requiring intensive care unit and mechanical ventilation were excluded. Therefore, our results cannot be extrapolated to unstable COPD exacerbations. Additionally, it was suggested that PCT is a specific biomarker for bacterial infections, more than CRP. However, PCT-guided strategies are relatively expensive, whereas CRP is cheap and widely available. Hence, cost-effectiveness comparisons are significant when comparing PCT and CRP-guided antibiotic strategies. Further, it could be argued that the patients conditions’ included in this study were not severe enough to require antibiotic therapy; this explains the lack of difference observed between two strategies in this study. Notably, however, all our patients were below the type 1 or 2 of the Anthonisen classification. Moreover, most patients had high CRP levels at their inclusion. Lastly, due to the relatively limited data regarding the optimal cutoff values that should be used in CRP-guided algorithms, it is not possible to anticipate whether different cutoffs or algorithms will be associated with different results.

## Conclusion

Our study showed that a 2-day course of levofloxacin was not inferior to a CRP-guided strategy, but exposes to a less antibiotic consumption.

## Supporting information

S1 File Consort checklist. (DOC)

S2 File (RAR)
